The article "Cardioprotective Mechanism and Active Compounds of Folium Ginkgo on Adriamycin-Induced Cardiotoxicity: A Network Pharmacology Study" was published in 2022. Journal: Comput Math Methods Med.

# Cardioprotective Mechanism and Active Compounds of *Folium Ginkgo* on Adriamycin-Induced Cardiotoxicity: A Network Pharmacology Study

**DOI:** 10.1155/2022/4338260

**Published:** 2022-09-28

**Authors:** Xue Sun, Yiming Zhu, Fang Li, Min Li, Guoxing Wan

**Affiliations:** ^1^Department of Oncology, Renmin Hospital, Hubei University of Medicine, 39# Chaoyang Road, Shiyan, Hubei 442000, China; ^2^Institute of Cancer, Renmin Hospital of Hubei University of Medicine, Shiyan 442000, China

## Abstract

**Objective:**

To investigate the mechanism of *Folium Ginkgo* (FG) against adriamycin-induced cardiotoxicity (AIC) through a network pharmacology approach.

**Methods:**

Active ingredients of FG were screened by TCMSP, and the targets of active ingredient were collected by Genclip3 and HERB databases. AIC-related target genes were predicted by Genecards, OMIM, and CTD databases. Protein-protein interaction (PPI) network was constructed by STRING platform and imported into Cytoscape software to construct the FG-active ingredients-targets-AIC network, and CytoNCA plug-in was used to analyze and identify the core target genes. The Metascape platform was used for transcription factor, GO and signaling pathway enrichment analysis.

**Results:**

27 active ingredients of FG and 1846 potential targets were obtained and 358 AIC target genes were retrieved. The intersection of FG and AIC targets resulted in 218 target genes involved in FG action. The top 5 active ingredients with most targets were quercetin, luteolin, kaempferol, isorhamnetin, and sesamin. After constructing the FG-active ingredients-targets-AIC network, CytoNCA analysis yielded 51 core targets, of which the top ranked target was STAT3. Ninety important transcription factors were enriched by transcription factor enrichment analysis, including RELA, TP53, NFKB1, SP1, JUN, STAT3, etc. The results of GO enrichment analysis showed that the effective active ingredient targets of FG were involved in apoptotic signaling, response to growth factor, cellular response to chemical stress, reactive oxygen species metabolic process, etc. The signaling pathway enrichment analysis showed that there were many signaling pathways involved in AIC, mainly including pathways in cancer, FOXO signaling pathway, AGE-RAGE signaling pathway in diabetic complications, signaling by interleukins, and PI3K-AKT signaling pathway,.

**Conclusions:**

The study based on a network pharmacology approach demonstrates that the possible mechanisms of FG against AIC are the involvement of multicomponents, multitargets, and multipathways, and STAT3 may be a key target. Further experiments are needed to verify the results.

## 1. Introduction

Adriamycin is a broad-spectrum, highly effective anthracycline antitumor drug that can be used in the treatment of a variety of solid and hematologic malignancies, especially important in the treatment of breast cancer, sarcoma, lymphoma, leukemia, and other cancers. However, the time- and dose-dependent cardiotoxicity caused by adriamycin has severely limited its clinical application and therapeutic efficacy. Adriamycin-induced cardiotoxicity (AIC) is observed at a wide range of 3%-48% in adult and can manifest as both acute irreversible myocardial injury, left ventricular dysfunction, dilated cardiomyopathy, and heart failure one or more years after the end of treatment [1]. Although current evidence indicates that AIC is associated with oxidative stress, mitochondrial damage, topoisomerase-2, intracellular environmental imbalance, cellular autophagy, and apoptosis, the exact mechanism remains unknown [2]. Dexrazoxane is the only drug recommended by current guidelines to mitigate AIC, however, the efficacy is limited [3]. Therefore, it is clinically important to explore effective therapeutic drugs to alleviate AIC.

*Folium Ginkgo* (FG) is the dried leaf of *Ginkgo biloba*, a plant of the Ginkgo family, which is naturally mild, with a slight air, slightly sweet, bitter, and astringent taste. FG has the effects of activating blood circulation, relieving pain, comforting the lungs and asthma, and reducing lipids, thus has been used in China as a traditional medicine for the treatment of asthma, bronchitis, and heart dysfunction for at least 5000 years [4, 5]. Modern pharmacological research has found that FG extract contains a variety of medicinal active ingredients, mainly including flavone glycosides, terpene lactones, ginkgolic acids, etc [6]. These active ingredients are the material basis for its anti-inflammatory, anti-polymerization, lipid-regulating, antioxidant, mitochondrial function protection, and cancer cell apoptosis promotion [7, 8]. The protective effects of FG extract on ventricular myocardial hypertrophy, postinfarction myocardial fibrosis, and ischemia-reperfusion myocardial injury in rats were reported by previous in-vivo studies [9]. Clinical studies have also found significant effects of FG extract in the treatment of coronary heart disease, stroke, angina pectoris, and other cardiovascular diseases [9, 10]. In addition to the wide use for cardio-cerebro-vascular diseases, previous study found its myocardial protection effect on cardiomyopathy as well [11]. Studies on the intervention of FG extracts against AIC have also been reported, demonstrating a better therapeutic effect [12]. Nevertheless, the molecular mechanism of FG extract against AIC is still unclear due to its complex composition and diverse targets. Network pharmacology which integrates systems biology and pharmacology, was widely used to explore the comprehensive mechanism of Chinese herbal medicine. As an effective and rapid tool, network pharmacology takes advantage of its capability in the aspect of elucidating the multitargets and multipathway mechanism to advance the drug discovery [13]. Therefore, this study adopted a network pharmacology approach to screen the active ingredients of FG and establish a disease-target-herbal medicine multilevel network to systematically investigate the possible mechanisms of FG against AIC and provide theoretical references for the development of drugs against AIC.

## 2. Materials and Methods

### 2.1. Screening of Active Ingredients and Targets of FG

The TCMSP database (https://tcmspw.com/tcmsp.php) was searched for the chemical composition of FG using “*Folium Ginkgo*” as the keyword. The possible active ingredients in FG were screened with an oral bioavailability (OB) ≥ 30% and drug-likeness (DL) ≥ 0.18, and the pharmacologic targets involved were identified. At the same time, using the screened active ingredients as keywords, the online tools Genclip3 (http://ci.smu.edu.cn/genclip3/analysis.php) and HERB (http://herb.ac.cn/) databases were used to further collect additional FG targets, and bioDBnet (https://biodbnet-abcc.ncifcrf.gov/db/db2db.php) was used to perform ID conversion of identified target gene. Finally, the results were summarized and organized to form the FG-targets database.

### 2.2. Target Screening of AIC

The targets related to AIC were obtained by searching the Genecards database (https://www.genecards.org), the human Mendelian genetic database (OMIM, https://omim.org/) and CTD (http://ctdbase.org/). After removing duplicate targets, gene names of targets were normalized and converted to gene ID by bioDBnet (https://biodbnet-abcc.ncifcrf.gov/db/db2db.php) to obtain the disease targets.

### 2.3. Network Construction of FG-Active Ingredient-Target-AIC

The active ingredient targets of FG were compared with the cardiotoxicity targets of anthracycline, and the common targets were screened using the venn diagram tool. The above obtained active ingredients of FG and common targets with AIC were collated, and the Cytoscape 3.7.2 software was used to construct the FG-active ingredients-targets-disease network.

### 2.4. Network Construction of Protein-Protein Interactions(PPIs) and Core Targets

The obtained common targets were imported into the STRING database (https://string-db.org/) to obtain the PPI network file. The species was selected as “Homo sapiens”, the interaction score parameter was set to 0.900, and the remaining were set as default. The “TSV” network file was obtained by removing the targets that did not interact with other proteins. The “TSV” file was imported into Cytoscape software, and the topological parameters of each target of the PPI network were analyzed by CytoNCA plug-in, and organized in an excel table, with the following parameters: betweenness, closeness, degree, local average connectivity (LAC), network centrality, and eigenvector. The median values of these six indicators were calculated separately, and the targets were identified as the core targets when all six indicators of the targets were greater than the median value. Subsequently, the core target network was constructed by Cytoscape software.

### 2.5. Enrichment Analysis of Gene Ontology, Transcription Factor and Signal Pathway

The core target genes obtained above were imported into the online tool Metascape (https://metascape.org/gp/index.html#/main/step1) to perform gene ontology (GO), transcription factor, and signaling pathway enrichment analysis, with the species setting as “H. sapiens” and the module setting as “Express Analysis”.

## 3. Results

### 3.1. Active Ingredients and Targets of FG

A total of 27 active ingredients were obtained after screening through the TCMSP database, including white fruit lactone, luteolin, quercetin, geranylin, lignan, etc. The basic information is shown in Table 1. The gene names of potential targets corresponding to each active ingredient were normalized, and a total of 1846 potential targets were obtained after removing duplicate targets (no corresponding target for luteolin).

### 3.2. AIC-Associated Targets

After searching for AIC target genes in Genecards, OMIM, and CTD databases, normalizing gene names and removing duplicate target genes, a total of 358 target genes were obtained.

### 3.3. FG-Active Ingredient-Target-AIC Network

The potential targets of the 27 active ingredients of FG were intersected with the target genes of AIC by the online venn diagram tool, resulting in 218 target genes (Figure 1), which indicated that these 218 targets were considered as potential targets of FG against AIC. The active ingredients of FG and their common targets with AIC were imported into Cytoscape 3.7.2 software to generate a FG-active ingredients-target-AIC network, as shown in Figure 2, where the common targets were in blue and the potential targets corresponding to the active ingredients in FG were in green. Figure 2 reflected that 27 active ingredients of FG might interfere with AIC through 218 potential targets. Among them, the top 5 active ingredients with most potential targets were quercetin (MOL000098, 191 targets), lignan (MOL000006, 146 targets), kaempferol (MOL000422, 120 targets), isorhamnetin (MOL000354, 76 targets), and sesquiterpene (MOL001558, 62 targets).

### 3.4. PPIs and Core Target Networks

The 218 common targets were imported into the STRING database to obtain the TSV network file of PPIs with high confidence, which were then imported into Cytoscape 3.7.2 software and analyzed by CytoNCA plug-in. According to the established criterion, 51 genes were identified as core targets, with which the PPI network was constructed as Figure 3. The topological characteristics of these 51 core targets were shown in Table 2, from which it could be seen that the target with best performance in all parameters was STAT3.

### 3.5. Enrichment Analysis Results

The 51 core target genes were imported into Metascape online software for enrichment analysis. Using *p* < 0.01 as the threshold, the results of transcription factor enrichment analysis showed that a total of 90 transcription factors were enriched, of which the top 20 were shown in Figure 4, including RELA, TP53, NFKB1, SP1, JUN, STAT3, and other transcription factors, which were considered to be the most important transcription factors involved in FG against AIC. Similarly, the top 20 GO and signaling pathway enrichment analyses were shown in Figures 5(a) and 5(b), including GO entries for apoptosis, growth factor stimulation response and cellular response to chemical stress and reactive oxygen metabolic processes, and signaling pathways such as cancer-related signaling pathway, FOXO signaling pathway, AGE-RAGE signaling pathway in diabetic complications, interleukin signaling pathway, and PI3K-AKT signaling pathway, which were considered to be the most important biological processes and signaling pathways involved in FG against AIC.

## 4. Discussion

Chemotherapy-induced cardiotoxicity is classified as “drug toxicity” in traditional Chinese medicine (TCM), of which anthracyclines are highly toxic. Therefore, patients receiving anthracycline chemotherapy often impair their vital energy with clinical symptoms including palpitations, chest tightness, shortness of breath, and weakness [14, 15]. Studies of TCM syndromes and syndrome elements suggest that the cardiotoxicity syndrome of anthracyclines is characterized by combination of deficiency and abundance, and the pathogenesis includes deficiency, dampness, stasis, and Qi-stagnation. “Deficiency” is the root of the disease, and “tonifying deficiency” is the basic treatment in the practice of TCM, with benefiting Qi and nourishing Yin, invigorating blood and resolving blood stasis as the main treatment method [16].

FG is a common Chinese medicine with the efficacy of activating blood circulation and removing blood stasis. A large number of basic and clinical studies have revealed a wide range of therapeutic effects of FG extract on cardiovascular and cerebrovascular diseases [9]. FG has also shown great potential in the prevention and treatment of AIC. Xu et al. found that FG extract was able to improve cardiac function and myocardial energy metabolism in rats experiencing AIC, and further studies showed that the mechanism may be associated with the increased expression of ghrelin peptide [17]. Li et al. also showed that FG extract could treat anthracycline-induced cardiomyopathy [12]. Ding et al. found that FG extract (EGb761) could antagonize AIC in rats without affecting its antitumor activity [18]. Similarly, the cardioprotective effect of FG extract (EGb761) reducing anthracycline-induced oxidative stress and apoptosis in rat and mouse cardiomyocytes was also confirmed by both in vivo and in vitro studies [19–24]. Nevertheless, FG extracts are mixtures containing multiple compounds with diverse targets, and the mechanisms of action often involve multiple signaling pathways. Therefore, even for the standardized FG extract EGb761 (containing 24% ginkgolide and 6% terpene lactone), the several studies to explore its anti-anthracycline cardiotoxicity are mostly concentered on phenotypic exploration, the specific mechanism of action remains to be further investigated.

Unlike the traditional “single compound-disease” approach, network pharmacology is suitable for studying the multiple components and mechanisms of action of TCM from a holistic perspective [25]. Therefore, this study was conducted to investigate the mechanism of action of FG on AIC using a network pharmacology approach. The results of this study showed that a total of 27 candidate active ingredients of FG were screened by TCMSP, most of which were flavonol glycosides, indicating that the main components of FG against AIC may rely on flavonol glycosides. Of the candidate active ingredients, the five with most targets were quercetin, lignan, kaempferol, isorhamnetin, and sesquiterpene. Moreover, 218 potential targets of AIC were also predicted. According to several studies, quercetin can improve myocardial energy metabolism, inhibit oxidative stress, improve myocardial mitochondrial function, and reduce myocardial apoptosis in rats, thus antagonizing AIC [26–28]. Studies on lignocaine, kaempferol, isorhamnetin, and sesquiterpene also showed cardioprotective effects against AIC [29–32]. Therefore, it was hypothesized that quercetin, lignan, kaempferol, isorhamnetin, and sesquiterpene might play important roles in the pharmacological mechanism of FG against AIC. In addition, 51 core targets were identified by PPI network analysis. Meanwhile, transcription factor enrichment analysis was performed on these core targets, resulting in 90 potentially important transcription factors, the top 20 of which were illustrated in Figure 4, including RELA, TP53, NFKB1, SP1, JUN, STAT3, etc. Notably, STAT3 was both one of the most important genes in the core target and one of the most important transcription factors enriched. Previous study has shown that inactivation of the JAK2/STAT3 signaling pathway significantly reduced myocardial reactive oxygen species and lipid oxidation levels, inhibited myocardial apoptosis and fibrosis, and promoted autophagy, thereby antagonizing AIC [33, 34], and FG extract was found able to suppress STAT3-mediated inflammatory signal in heart, brain, and liver tissue for protection purpose [35–37], implying that STAT3 may be an important target for FG to treat AIC.

The results of GO enrichment analysis showed that the active ingredients of FG are involved in biological processes such as apoptosis, growth factor stimulation response, and cellular response to chemical stress and reactive oxygen metabolic processes, suggesting that the targets of FG are involved in apoptosis and oxidative stress regulation. Signaling pathway enrichment analysis showed that numerous signaling pathways, including cancer-related signaling pathway, Foxo signaling pathway, AGE- RAGE signaling pathway in diabetic complications, interleukin signaling pathway, and PI3K-AKT signaling pathway were involved in the mechanism of FG against AIC. Among them, as a classical pathways to maintain cell survival cycle, activation of PI3K-AKT signaling was demonstrated to effectively attenuate myocardial apoptosis and fibrosis induced by anthracycline [38–40]. Consistently, the therapeutic effect of FG active ingredients ginkgolide A, ginkgolide B, and isorhamnetin has been recently validated via their synergistic effect on PI3K-AKT activation in vitro [12]. Interleukin-mediated regulation of inflammation has an important role in anthracycline cardiotoxicity, and different interleukin signaling may play different roles. Previous studies have found that doxorubicin induces proinflammatory factor IL-1*β* overexpression and promotes myocardial inflammation and apoptosis through activation of NF-*κ*B signaling [41], while activating NF-*κ*B signaling accelerated doxorubicin-induced apoptosis and fibrosis in cardiac cells [42]. In support of this, FG has been also found to show a protective effect against AIC by inhibiting NF-*κ*B signaling [12], however, that whether this effect on NF-*κ*B was mediated by interleukin signaling remained unclear. Foxo signaling is important for the regulation of cardiomyocyte development and survival. Doxorubicin has been shown to induce cardiomyocyte apoptosis and atrophy through CDK2-mediated activation of FOXO1 signaling [43], while overexpression of Foxo3A attenuates AIC by inhibiting MIEF2 and mitochondrial disintegration in cardiomyocytes [44], and activation of FOXO3A signaling reduces anthracycline-induced apoptosis in rat cardiomyocytes [45], indicating the diversity of FOXO signal in cardiomyocytes. In addition, PI3K-AKT activation was found to upregulate FOXO3A signaling to antagonize AIC [46]. According to the results of the current study, STAT3, FOXO1, and FOXO3 are both the core targets of FG against AIC and the core genes in the aforementioned key signaling, suggesting that there may be synergistic effects among multiple targets and signaling pathways for FG in intervening AIC cardiotoxicity.

## 5. Conclusion

In summary, this study systematically investigated the active ingredients, targets, and signaling pathways of FG against AIC based on a network pharmacology approach. Quercetin, lignan, kaempferol, isorhamnetin, and sesquiterpene were identified as key components of FG in the treatment of AIC and STAT3 was identified as the key target. The synergistic effects of multiple ingredients, targets, and pathways may be implicated in FG action. Given the limitations of network pharmacology, further experimental validation of the effect of the key compounds of FG on important targets and signal such as STAT3 and FOXO signal AIC model is needed in the future, which could provide more support for our finding.

## Figures and Tables

**Figure 1:** Venn diagram of FG active ingredients and AIC targets. AIC, adriamycin-induced cardiotoxicity; FG, *Folium Ginkgo*.

**Figure 2:** FG-active ingredient-target-adriamycin cardiotoxicity network. AIC, adriamycin-induced cardiotoxicity; FG, *Folium Ginkgo;* common targets between *Ginkgo biloba* active ingredients and AIC in blue oval; *FG* active ingredient compounds and their numbers in green rectangles.

**Figure 3:** Core target networks of FG against AIC.

**Figure 4:** Enrichment analysis of transcription factor of core targets.

**Figure 5:** GO and signaling pathway enrichment analysis.

**Table 1:** Active ingredient of *Folium Ginkgo.*

Mol ID	Compounds	OB (%)	DL
MOL011578	Bilobalide	84.42	0.36
MOL002680	Flavoxanthin	60.41	0.56
MOL001558	Sesamin	56.55	0.83
MOL000492	(+)-Catechin	54.83	0.24
MOL000096	(-)-Catechin	49.68	0.24
MOL000354	Isorhamnetin	49.60	0.31
MOL011589	Ginkgolide M	49.09	0.75
MOL011587	Ginkgolide C	48.33	0.73
MOL000098	Quercetin	46.43	0.28
MOL007179	Linolenic acid ethyl ester	46.10	0.20
MOL011588	Ginkgolide J	44.84	0.74
MOL011586	Ginkgolide B	44.38	0.73
MOL000449	Stigmasterol	43.83	0.76
MOL001490	Bis[(2S)-2-ethylhexyl] benzene-1,2-dicarboxylate	43.59	0.35
MOL001494	Mandenol	42.00	0.19
MOL011597	Luteolin-4′-glucoside	41.97	0.79
MOL000422	Kaempferol	41.88	0.24
MOL011594	Isogoycyrol	40.36	0.83
MOL005043	Campest-5-en-3beta-ol	37.58	0.71
MOL005573	Genkwanin	37.13	0.24
MOL000358	Beta-Sitosterol	36.91	0.75
MOL011604	Syringetin	36.82	0.37
MOL000006	Luteolin	36.16	0.25
MOL003044	Chryseriol	35.85	0.27
MOL009278	Laricitrin	35.38	0.34
MOL002883	Ethyl oleate	32.40	0.19
MOL002881	Diosmetin	31.14	0.27

OB, oral bioavailability; DL, drug-likeness.

**Table 2:** Topological parameters of FG-active ingredient-target-AIC network.

Gene	Betweenness	Closeness	Degree	Eigenvector	LAC	NC
STAT3	3613.524	0.141538	41	0.25225	8.487805	25.03794
HSP90AA1	4155.85	0.140673	38	0.216973	6.210526	16.68387
TP53	3109.456	0.139924	36	0.202642	6.722222	18.50258
AKT1	3549.988	0.14143	36	0.225162	7.666667	19.34911
SRC	2349.084	0.139288	35	0.221844	8.057143	19.30701
MAPK1	2233.733	0.140888	35	0.217537	6.857143	16.91455
EP300	3296.193	0.140673	33	0.196503	7.151515	16.27721
PIK3CA	1124.138	0.136600	31	0.188837	6.451613	16.56008
ESR1	927.866	0.139394	27	0.220745	9.851852	15.0709
EGFR	622.7751	0.136803	26	0.193300	8.538462	14.81648
CTNNB1	861.7669	0.137519	25	0.184046	7.360000	11.47712
FOXO3	1100.573	0.137519	25	0.172923	7.520000	13.81911
FOS	1658.016	0.137519	24	0.166604	6.750000	10.6718
MYC	612.8622	0.13845	23	0.184177	8.695652	12.46751
FOXO1	1242.73	0.136499	22	0.144507	6.272727	11.44315
CAV1	957.2685	0.136803	20	0.134328	4.800000	6.392411
HIF1A	247.0885	0.137007	20	0.177245	9.100000	12.04197
MAPK8	780.4704	0.136397	19	0.119740	3.789474	5.508794
RAC1	374.3938	0.135294	19	0.152714	7.263158	9.57265
EDN1	988.8267	0.136095	19	0.128492	5.052632	6.761953
MAPK14	480.6648	0.137416	19	0.153469	6.736842	7.919192
VEGFA	603.2804	0.135195	19	0.141028	6.421053	8.723443
TNF	851.584	0.134897	19	0.093954	4.421053	7.889854
RXRA	2372.955	0.137007	18	0.086172	3.333333	7.43355
EGF	511.6375	0.134209	17	0.126609	6.352941	8.987879
MDM2	193.1254	0.134405	14	0.103356	5.428571	6.945177
CXCR4	274.9352	0.132279	14	0.086078	4.571429	6.542025
PPARA	1177.08	0.135693	13	0.072716	3.846154	6.213203
CASP3	669.0858	0.132374	13	0.071404	2.461538	4.450000
AGT	1014.253	0.131994	12	0.060731	2.666667	5.11039
BCL2	691.7133	0.135095	12	0.091332	4.666667	6.916667
INS	808.0313	0.131617	12	0.075362	2.833333	3.336364
IL1B	341.9638	0.13343	12	0.063619	3.833333	4.931061
ABL1	104.5201	0.131241	11	0.078031	3.818182	4.838095
CXCL8	166.0439	0.132184	11	0.058389	4.545455	5.835714
PTEN	250.5796	0.131805	11	0.083429	4.000000	4.933333
IL2	498.0181	0.133624	11	0.086090	3.454545	4.725000
IGF1	77.82508	0.130127	11	0.091381	5.090909	5.722222
CDK2	74.20501	0.130035	10	0.069160	4.600000	6.023810
CAT	1212.973	0.129852	10	0.035067	2.400000	4.611111
MMP2	204.2059	0.131148	10	0.064443	3.600000	5.238095
BRCA1	415.0989	0.130868	9	0.065461	3.777778	4.928571
CSF2	79.61738	0.130127	9	0.056202	4.000000	5.375000
ATM	49.85902	0.129944	8	0.051793	4.250000	5.428571
ADRBK1	262.6582	0.129123	8	0.038637	2.500000	2.952381
HSPA1A	222.7726	0.132852	8	0.054802	2.750000	3.761905
POMC	527.4912	0.127336	8	0.036912	2.500000	3.657143
FGFR3	69.17835	0.132565	8	0.074942	4.500000	6000000
BAX	166.4043	0.128942	7	0.038510	2.857143	4.250000
MCL1	57.92171	0.13266	7	0.061129	3.428571	4.000000
SOD2	327.0613	0.128045	7	0.034584	3.142857	4.566667

LAC, local average connectivity; NC, network centrality.

## Data Availability

The data used to support the findings of this study are all included within the article.

## References

[1] Sangweni N. F., van Vuuren D., Mabasa L. (2022). Prevention of anthracycline-induced cardiotoxicity: the good and bad of current and alternative therapies. *Frontiers in Cardiovascular Medicine*.

[2] Rawat P. S., Jaiswal A., Khurana A., Bhatti J. S., Navik U. (2021). Doxorubicin-induced cardiotoxicity: an update on the molecular mechanism and novel therapeutic strategies for effective management. *Biomedicine & Pharmacotherapy*.

[3] Varghese S. S., Eekhoudt C. R., Jassal D. S. (2021). Mechanisms of anthracycline-mediated cardiotoxicity and preventative strategies in women with breast cancer. *Molecular and Cellular Biochemistry*.

[4] Qian Y. Y., Zhu G. Q., Wang W. J., Gao Q. (2021). Advances in the clinical and pharmacological effects of ginkgolides and their preparations. *Chinese Traditional Patent Medicine*.

[5] Birks J., Grimley E. J. (2009). Ginkgo biloba for cognitive impairment and dementia. *Cochrane Database of Systematic Reviews*.

[6] Zuo W., Yan F., Zhang B., Li J., Mei D. (2017). Advances in the studies of Ginkgo biloba leaves extract on aging-related diseases. *Aging and Disease*.

[7] Yuan L., Li Y., Xu Z. M., Wen X. D., Li P. (2019). Research progress of *Ginkgo biloba* extracts for the treatment of ischemic stroke. *Progress in Pharmaceutical Sciences*.

[8] Liu Y., Xin H., Zhang Y., Che F., Shen N., Cui Y. (2022). Leaves, seeds and exocarp of *Ginkgo biloba* L . (Ginkgoaceae): a comprehensive review of traditional uses, phytochemistry, pharmacology, resource utilization and toxicity. *Journal of Ethnopharmacology*.

[9] China Physicians Association Integrative Medicine Physicians Section, National Clinical Medical Research Center of Chinese Medicine for Cardiovascular Diseases and Cardiovascular Disease Project Group of China Center for Evidence-Based Chinese Medicine (2020). Chinese expert consensus on the clinical application of oral *Ginkgo biloba* preparations (2020). *Chinese Journal of Integrated Traditional and Western Medicine*.

[10] Wang Q. L., Zhang M. X., Wang Q. L., Guo X. D. (2021). Research progress on the mechanism of Ginkgo biloba extracts against inner ear diseases. *Chinese Traditional Patent Medicine*.

[11] Shaito A., Thuan D., Phu H. T. (2020). Herbal medicine for cardiovascular diseases: efficacy, mechanisms, and safety. *Frontiers in Pharmacology*.

[12] Li Y., Xu C., Wang H. (2021). Systems pharmacology reveals the multi-level synergetic mechanism of action of *Ginkgo biloba L.* leaves for cardiomyopathy treatment. *Journal of Ethnopharmacology*.

[13] Nogales C., Mamdouh Z. M., List M., Kiel C., Casas A. I., Schmidt H. (2022). Network pharmacology: curing causal mechanisms instead of treating symptoms. *Trends in Pharmacological Sciences*.

[14] Guo S. L., Qiao Y. X., Yu M., Xue Y. T. (2021). Research progress on Chinese medicine to prevent cardiotoxicity of chemotherapy drugs. *Acta Chinese Medicine*.

[15] Jiang Y. P., Lin Z. C., Lin D. Z., Liu L., Wang H. Q. (2019). Chinese medicine treatment of anthracycline-induced cardiotoxicity from the "positive and negative view" of Huangdi Neijing. *Lishizhen Medicine and Materia Medica Research*.

[16] Yang H. F., Huang P. N., Liu Z. H., Liu A. P. (2020). A preliminary study on TCM syndromes and syndrome elements of anthracyclines acute cardiotoxicity. *Journal of Emergency in Traditional Chinese Medicine*.

[17] Xu Z. W., Wu W. K., Lan T. H., Zhang X. H. (2009). Protective effects of extract of *Ginkgo biloba* on adriamycin-induced heart failure and its mechanism: role of ghrelin peptide. *China Journal of Chinese Materia Medica*.

[18] Ding Q. X., Liu G. T. (1999). Protection of *Ginkgo biloba* extract (EGb761) against doxorubicin- induced cardiotoxicity without interfering with its antitumor activity. *Chinese Pharmaceutical Journal*.

[19] Boghdady N. A. (2013). Antioxidant and antiapoptotic effects of proanthocyanidin and Ginkgo biloba extract against doxorubicin-induced cardiac injury in rats. *Cell Biochemistry and Function*.

[20] Liu T. J., Yeh Y. C., Ting C. T. (2008). Ginkgo biloba extract 761 reduces doxorubicin-induced apoptotic damage in rat hearts and neonatal cardiomyocytes. *Cardiovascular Research*.

[21] Jasim S. T., Al-Kuraishy H. M., Al-Gareeb A. I. (2019). Gingko Biloba protects cardiomyocytes against acute doxorubicin induced cardiotoxicity by suppressing oxidative stress. *Journal of Pakistan Medical Association*.

[22] El-Boghdady N. A. (2013). Increased cardiac endothelin-1 and nitric oxide in adriamycin-induced acute cardiotoxicity: protective effect of Ginkgo biloba extract. *Indian Journal of Biochemistry & Biophysics*.

[23] Naidu M. U., Kumar K. V., Mohan I. K., Sundaram C., Singh S. (2002). Protective effect of Gingko biloba extract against doxorubicin-induced cardiotoxicity in mice. *Indian Journal of Experimental Biology*.

[24] Timioglu O., Kutsal S., Ozkur M. (1999). The effect of EGb 761 on the doxorubicin cardiomyopathy. *Research Communications in Molecular Pathology and Pharmacology*.

[25] Chu M., He R., Pang H. S., Hu F. Y. (2021). The molecular targets and therapeutic mechanisms of Er Miao san treating atopic dermatitis based on network pharmacology. *International Journal of Traditional Chinese Medicine*.

[26] Chen X., Peng X., Luo Y. (2019). Quercetin protects cardiomyocytes against doxorubicin-induced toxicity by suppressing oxidative stress and improving mitochondrial functionvia14-3-3*γ*. *Toxicology Mechanisms and Methods*.

[27] Zakaria N., Khalil S. R., Awad A., Khairy G. M. (2018). Quercetin reverses altered energy metabolism in the heart of rats receiving Adriamycin chemotherapy. *Cardiovascular Toxicology*.

[28] Sharma A., Parikh M., Shah H., Gandhi T. (2020). Modulation of Nrf2 by quercetin in doxorubicin-treated rats. *Heliyon*.

[29] Zhang Y., Ma C., Liu C., Wei F. (2020). Luteolin attenuates doxorubicin-induced cardiotoxicity by modulating the PHLPP1/AKT/Bcl-2 signalling pathway. *PeerJ*.

[30] Xiao J., Sun G. B., Sun B. (2012). Kaempferol protects against doxorubicin-induced cardiotoxicity *in vivo* and *in vitro*. *Toxicology*.

[31] Sun J., Sun G., Meng X. (2013). Isorhamnetin protects against doxorubicin-induced cardiotoxicity in vivo and in vitro. *PLoS One*.

[32] Su S., Li Q., Liu Y. (2014). Sesamin ameliorates doxorubicin-induced cardiotoxicity: involvement of Sirt1 and Mn-SOD pathway. *Toxicology Letters*.

[33] Rong J., Li L., Jing L., Fang H., Peng S. (2016). JAK2/STAT3 pathway mediates protection of metallothionein against doxorubicin-induced cytotoxicity in mouse cardiomyocytes. *International Journal of Toxicology*.

[34] Zhang J., Sun Z., Lin N. (2020). Fucoidan from *Fucus vesiculosus* attenuates doxorubicin-induced acute cardiotoxicity by regulating JAK2/STAT3-mediated apoptosis and autophagy. *Biomedicine & Pharmacotherapy*.

[35] Zhang Y., Liu J., Yang B. (2018). Ginkgo biloba extract inhibits astrocytic lipocalin-2 expression and alleviates neuroinflammatory injury via the JAK2/STAT3 pathway after ischemic brain stroke. *Frontiers in Pharmacology*.

[36] Sherif I. O., Al-Shaalan N. H. (2022). Hepatoprotective effect of Ginkgo biloba extract against methotrexate-induced hepatotoxicity via targeting STAT3/miRNA-21 axis. *Drug and Chemical Toxicology*.

[37] Li Y., Xiong Y., Zhang H. (2017). Ginkgo biloba extract EGb761 attenuates brain death-induced renal injury by inhibiting pro-inflammatory cytokines and the SAPK and JAK-STAT signalings. *Scientific Reports*.

[38] Li X., Zhong J., Zeng Z. (2020). MiR-181c protects cardiomyocyte injury by preventing cell apoptosis through PI3K/Akt signaling pathway. *Cardiovascular Diagnosis and Therapy*.

[39] Nie L., Liu M., Chen J. (2021). Hydrogen sulfide ameliorates doxorubicin- induced myocardial fibrosis in rats via the PI3K/AKT/mTOR pathway. *Molecular Medicine Reports*.

[40] Alzahrani A. M., Rajendran P., Veeraraghavan V. P., Hanieh H. (2021). Cardiac protective effect of Kirenol against doxorubicin-induced cardiac hypertrophy in H9c2 cells through Nrf2 signaling via PI3K/AKT pathways. *International Journal of Molecular Sciences*.

[41] Peng W., Rao D., Zhang M. (2020). Teneligliptin prevents doxorubicin-induced inflammation and apoptosis in H9c2 cells. *Archives of Biochemistry and Biophysics*.

[42] Wang Z. Q., Chen M. T., Zhang R., Zhang Y., Li W., Li Y. G. (2016). Docosahexaenoic acid attenuates doxorubicin-induced cytotoxicity and inflammation by suppressing NF-*κ*B/iNOS/NO signaling pathway activation in H9C2 cardiac cells. *Journal of Cardiovascular Pharmacology*.

[43] Xia P., Chen J., Liu Y., Fletcher M., Jensen B. C., Cheng Z. (2020). Doxorubicin induces cardiomyocyte apoptosis and atrophy through cyclin- dependent kinase 2-mediated activation of forkhead box O1. *The Journal of Biological Chemistry*.

[44] Zhou L., Li R., Liu C. (2017). Foxo3a inhibits mitochondrial fission and protects against doxorubicin-induced cardiotoxicity by suppressing MIEF2. *Free Radical Biology & Medicine*.

[45] Zhang X., Li J., Cheng Y., Yi J., Liu X., Cheng W. (2018). Downregulation of CUEDC2 prevents doxorubicin-induced cardiotoxicity in H9c2 cells. *Molecular Medicine Reports*.

[46] Liu M. H., Zhang Y., He J. (2016). Hydrogen sulfide protects H9c2 cardiac cells against doxorubicin-induced cytotoxicity through the PI3K/Akt/FoxO3a pathway. *International Journal of Molecular Medicine*.

